# The Therapeutic Effects of Extracorporeal Shock Wave Therapy (ESWT) on the Rotator Cuff Lesions with Shoulder Stiffness: A Prospective Randomized Study

**DOI:** 10.1155/2020/6501714

**Published:** 2020-05-13

**Authors:** Jih-Yang Ko, Kai-Kit Siu, Feng-Sheng Wang, Ching-Jen Wang, Wen-Yi Chou, Chung-Cheng Huang, Shu-Jui Kuo

**Affiliations:** ^1^Department of Orthopedic Surgery, Kaohsiung Chang Gung Memorial Hospital, Kaohsiung, Taiwan; ^2^Department of Medical Research, Kaohsiung Chang Gung Memorial Hospital, Kaohsiung, Taiwan; ^3^Center for Shockwave Medicine and Tissue Engineering, Kaohsiung Chang Gung Memorial Hospital, Kaohsiung, Taiwan; ^4^Department of Orthopedic Surgery, Xiamen Chang Gung Hospital, Xiamen, China; ^5^Core Laboratory for Phenomics and Diagnostics, Kaohsiung Chang Gung Memorial Hospital, Kaohsiung, Taiwan; ^6^Department of Radiology, Kaohsiung Chang Gung Memorial Hospital, Kaohsiung, Taiwan; ^7^School of Medicine, China Medical University, Taichung, Taiwan; ^8^Department of Orthopedic Surgery, China Medical University Hospital, Taichung, Taiwan

## Abstract

**Aim:**

We wish to investigate the therapeutic potential of a single-session high-energy extracorporeal shock wave therapy (ESWT) on the rotator cuff lesions with shoulder stiffness. *Patients and Methods*. Thirty-seven patients afflicted with rotator cuff lesions with shoulder stiffness were randomized to receive either shockwave or sham treatment based on statistical randomization. In the shockwave group, we used Orthospec™ Extracorporeal Shock Wave Therapy 3000 impulse 24 kV (0.32 mJ/mm^2^) focused at two points as one session. The sham intervention entailed the use of the device in which the silicone pad was removed from the stand-off device. The visual analogue scale (VAS), muscle power of the shoulder, Constant and Murley score (CMS), and range of motion (ROM) of the shoulder were assessed for all patients. Ten milliliters of peripheral venous blood was obtained from every participant for the measurements of markers for inflammation, tissue regeneration, angiogenesis, and substance P before and at 1 week and 4 weeks after intervention.

**Results:**

The ESWT group has significantly better VAS, muscle power, CMS, and ROM at 6 and 12 months after intervention. No between-group differences were observed before as well as 1 and 4 weeks after intervention in the selected biomarkers.

**Conclusion:**

ESWT may be a good adjuvant for the treatment of rotator cuff lesions with shoulder stiffness.

## 1. Introduction

Shoulder stiffness is characterized by pain and loss of shoulder motion. Some patients have no identifiable cause (so-called “idiopathic adhesive capsulitis”), and others are caused by underlying diseases, especially rotator cuff lesions [1]. Rotator cuff lesions are the common shoulder disorder manifested by pain, limited motion, weakness, and functional disability. Intrinsic degeneration, outlet impingement, and inflammatory process are the important mechanisms underlying the pathogenesis of the rotator cuff lesions [2–5]. Increased expression of IL-1*β* and myofibroblast recruitment in the subacromial bursa in rotator cuff lesions could be observed in shoulder stiffness, suggesting that rotator cuff lesions with shoulder stiffness are an inflammatory disease [5]. Treatment options for shoulder stiffness include physical therapy, intra-articular corticosteroid injection, closed manipulation, and open or arthroscopic release [1, 6–10]. Faster improvement of the range of motion is desirable, and even the surgical repair of the rotator cuff lesions is needed later, underscoring the importance of an effective treatment for shoulder stiffness [2, 11–13]. However, none of the treatment alternatives is simple, effective, and noninvasive.

Extracorporeal shockwave therapy (ESWT) has been utilized in the treatment of shoulder disorders, such as calcific tendinitis, with favorable outcomes for more than 20 years [14–19]. Anti-inflammation has been proposed as the pivotal component for the therapeutic effects of ESWT [6].

Because of the inflammatory nature of the rotator cuff lesions with shoulder stiffness and the anti-inflammatory effects of ESWT, we performed a double-blinded, prospectively randomized study to ascertain our hypothesis that ESWT can exert therapeutic potentials on rotator cuff lesions with shoulder stiffness [20].

## 2. Materials and Methods

This prospective randomized double-blinded study was approved by the Institutional Review Board of Kaohsiung Chang Gung Memorial Hospital (IRB 101-1810A3), being performed between July 2014 and April 2017 to compare the effects of ESWT and sham intervention on the patients with rotator cuff lesions with shoulder stiffness. All experiments were performed in accordance with relevant guidelines and regulations. This study was registered in the ClinicalTrials.gov system (ID: NCT02450864) on April 13, 2015. Valid written informed consent was procured from every participant.

The minimum sample size required for each group was calculated by the G∗Power 3.1.9.2 software (http://www.gpower.hhu.de/en.html). Input parameters were as follows: “*t* test” for test family, which “means Wilcoxon-Mann-Whitney test (two groups)” for statistical test, and “a priori” for the type of power analysis. The sample size of at least 15 for each group was thus derived (effect size: 1; *α* level: 0.05; power: 80%; allocation ratio: 1).

Subjects were considered eligible if they had (1) pain (visual analogue scale > 3) and stiffness of the shoulder, in which shoulder stiffness was defined by loss of >50% range of motion in any direction or the sum of range of motion < 270°; (2) a positive impingement sign and/or pain with Hawkins' test; (3) positive imaging diagnosis of supraspinatus lesion without complete tear on magnetic resonance imaging (MRI); and (4) pain and stiffness which did not respond to activity modification and/or physiotherapy under therapists for at least 3 months and (5) were aged between 35 and 80 years. We excluded the patients with rheumatic diseases, glenohumeral osteoarthritis, full-thickness cuff tears, fractures, infections, neoplasms, pregnancy, and subacromial injection within 3 weeks and the subjects not submitting valid written informed consent.

The imaging diagnosis of supraspinatus lesion was established by magnetic resonance imaging (MRI). On MRI, supraspinatus tendinopathy was characterized by increased intratendinous signal intensity on T2-weighted images without tendon disruption. Partial thickness tear was characterized by the presence of focal hyperintense fluid or a fluid-like signal extending into the tendon substance on the T2-weighted images. A full thickness tear was diagnosed by the extension of hyperintense fluid or fluid-like signals through the entire tendon on T2-weighted images [3, 5, 11]. The imaging diagnosis of MRI was based upon the consensus between the orthopedic surgeon (1^st^ author) and the radiologist (6^th^ author).

The participants were randomized into 2 groups immediately before the intervention by the computer-generated randomization list concealed in a set of numbered envelopes. The research assistant blinded to the clinical information of the participants opened the concealed envelope, and the card inside indicated whether the patient was randomized to the ESWT or sham group. The participants and the follow-up examiners were all blinded to the treatment assignment. In the ESWT group, patients received 3000 impulses of shockwave at 24 kV (energy flux density, 0.32 mJ/mm^2^) to the affected shoulder at subacromial space and rotator interval in one session. Each session lasted for one hour. The source of the shockwaves was an Orthospec™ Extracorporeal Shockwave (Orthospec™- Medispec, Israel). ESWT was performed by a specialist certified for operating the machine on an outpatient basis. The area of treatment was clinically focused with a control guide on the machine, and surgical lubricant was placed on the skin in contact with the shockwave tube. Shockwaves were clinically focused at two areas. Area 1 is the subacromial area, about one finger breadth below the anterior lateral border of the acromion tip. Area 2 is the rotator interval, about one finger breadth lateral and above to the coracoid process. Local anesthetics were prohibited. The sham intervention entailed the use of the device in which the silicone pad was removed from the stand-off device, but the patients could still hear the sound of the shock wave and have tingling sensation over the skin but without energy transduced. The vital signs and any discomforts were monitored throughout the course of treatment. The treated areas were inspected for local swelling, ecchymosis, or hematoma after the treatment. Baseline activity modification and/or physiotherapy was sustained after the intervention. Gentle pendulum exercise as well as assisted shoulder elevation and external and internal rotation was initiated after intervention for all the participants. After treatment and during follow-ups, patients were restricted to the use of a 1000 mg of acetaminophen per day for pain, in order to facilitate the usage and comparison of the medications among the patients. Patients had a pain medication-free interval 3 days prior to each evaluation. Patients who had persistent and severe shoulder discomfort were advised to undergo surgical intervention.

The clinical parameters and serum biomarkers were assessed before and after intervention. The clinical parameters included visual analogue scale (VAS), muscle power for shoulder abduction, Constant and Murley score (CMS), and range of motion (ROM) of the shoulder. Visual analogue scale (VAS) is a scale used for pain measurement with 0 point indicating no pain and 10 points indicating unbearable pain. The muscle power for shoulder abduction was examined during the maximal isometric contraction of the abductor muscles using a handheld dynamometer in shoulder 45° abduction and elbow 90° flexion without torso stabilization [21, 22]. The Constant and Murley score (CMS) is a standardized scale of assessing shoulder function with a maximum score of 100 points with a higher score indicating better shoulder function [23]. The range of motion (ROM) of the shoulder was measured with the patient in a sitting position. A goniometer was used to measure the angle to which the patient could maximally passively forward flex or abduct the shoulder. External rotation and internal rotation of the shoulders were determined with the patient's arm in a resting position and in a 45° flexion position, respectively. Normal shoulder ROM without scapular stabilization was considered to be 180° of forward flexion, 180° of abduction, 90° of external rotation, and 90° of internal rotation. By summation of the measured ROM, the sum of range of motion (SROM) was obtained [12]. Shoulder stiffness was defined by loss of more than 50% of range of motion in any direction or the SROM < 270° [24]. The clinical parameters were assessed before and 1 week, 4 weeks, 3 months, 6 months, and 12 months after intervention. The serum biomarkers were also assessed for the systemic impact of the intervention. Ten milliliters of peripheral venous blood was obtained from every participant for the measurements of interleukin 6 (IL-6), tumor necrosis factor-alpha (TNF-*α*), interleukin 1-beta (IL-1*β*), transforming growth factor-beta 1 (TGF-*β*1) for inflammation, insulin-like growth factor-1 (IGF-1), dickkopf-related protein 1 (DKK-1) for tissue regeneration, vascular endothelial growth factor (VEGF) for angiogenesis, and substance P for pain threshold before and at 1 week and 4 weeks after intervention. The choice for the blood sampling time was based upon our previous publications [25].

The data are expressed as the median (lower quartile and upper quartile). Categorical variables were compared by chi-square testing. The Mann–Whitney *U* test compared differences between groups. The Friedman test was utilized for the repeated measure analysis of repeated within-group comparisons for continuous variables, and the Wilcoxon signed-rank test was used for post hoc analysis. All statistics were performed by SPSS software, and a *p* value of <0.05 was considered to be statistically significant [26].

## 3. Results

There were 41 patients assessed for eligibility. Two patients did not meet the inclusion criteria, and two failed to offer informed consent. The remaining 37 patients were randomized into two groups (Figure 1). There were no statistical differences in the demographic profiles between the two groups (Table 1). There were 8 (42.1%) and 4 (22.2%) patients who suffered from partial supraspinatus tear in the ESWT group and sham group, respectively (*p* = 0.197).

In the ESWT group (19 patients), two patients underwent rotator cuff repair surgeries due to persistent discomfort 4 weeks and 3 months after ESWT, respectively. One patient lost to follow-up 3 months after ESWT. The remaining 16 patients were followed up to 12 months after ESWT. In the sham group (18 patients), one shifted to rotator cuff repair surgery 1 week after treatment and two lost to follow-up 3 months after intervention. The remaining 15 patients were followed up to 12 months.

The baseline VAS (*p* = 0.807), muscle power (*p* = 0.089), and CMS (*p* = 0.470) were comparable between the two groups. The subjects receiving ESWT experienced substantially better VAS (*p* = 0.012), stronger muscle power (*p* = 0.034), and higher CMS (*p* = 0.026) 6 months after intervention. The VAS was 0.0 (0.0, 0.0) for the ESWT group and 0.5 (0.0, 2.0) for the sham group 12 months after intervention (*p* = 0.025). The muscle power was 20.0 lb (20.0, 22.3) for the ESWT group and 17.5 lb (16.0, 20.0) for the sham group 12 months after intervention (*p* = 0.002). The CMS was 91.5 (89.8. 95.0) for the ESWT group and 85.0 (72.0, 87.0) for the sham group 12 months after intervention (*p* = 0.005). In other words, the subjects receiving ESWT experienced better VAS, muscle power, and CMS 6 and 12 months after intervention (Table 2).

We also measured the range of motion (ROM) of forward flexion, abduction, external rotation, internal rotation, and sum of range of motion (SROM) between the two groups. The range of motion in all directions, including SROM, was comparable between the two groups before the intervention. The subjects receiving ESWT experienced better internal rotation 3 months after intervention (*p* = 0.039). The participants receiving ESWT experienced better external rotation (*p* = 0.012), internal rotation (*p* < 0.001), and SROM (*p* = 0.023) 6 months after intervention. The range of motion was 170.0° (165.0°, 175.0°) in forward flexion, 165.0° (160.0°, 170.0°) in abduction, 80.0° (68.8°, 81.3°) in external rotation, 70.0° (60.0°, 76.3°) in internal rotation, and 485.0° (457.5°, 502.5°) in SROM for the ESWT group 12 months after intervention. The range of motion was 162.5°(150.0°, 175.0°) in forward flexion, 150.0° (123.8°, 170.0°) in abduction, 70.0° (60.0°, 75.0°) in external rotation, 60.0° (51.3°, 70.0°) in internal rotation, and 445.0° (375.0°, 470.0°) in SROM for the sham group 12 months after intervention. Better forward flexion (*p* = 0.048), abduction (*p* = 0.009), external rotation (*p* = 0.042), internal rotation (*p* = 0.031), and SROM (*p* = 0.008) for the ESWT group were observed 12 months after intervention (Table 3).

The levels of serum biomarkers in baseline as well as in 1 and 4 weeks after intervention are summarized in Table 4. No between-group differences were observed before and 1 and 4 weeks after intervention.

Two patients in the ESWT group reported transient erythematous swelling at the treatment site (2 of 19, 10.5%). All of the symptoms subsided 1 to 2 days after ESWT. One patient (1 of 19, 5.26%) reported petechial bleeding at the treatment site which resolved spontaneously 1 week later. No complications have been observed in the sham group.

## 4. Discussion

Although rotator cuff lesions with shoulder stiffness have been previously described as a self-limiting process, recent reports have shown that it can lead to long-term disability [13, 27, 28]. There is no consensus concerning the treatment of rotator cuff lesions with shoulder stiffness at present. Physical therapy, intra-articular corticosteroid injections, closed manipulation, and open or arthroscopic release have been proposed, but none has been proven to be simple, effective, and noninvasive [1, 6–10].

The proposed mechanisms for ESWT include altering cellular activity through cavitation, blocking the gate control mechanism, altering cellular permeability, and enhancing angiogenesis, acoustic microstreaming, hyperstimulation of nociceptors, and anti-inflammatory and antifibrogenic effects [6, 17, 29–31]. Because shoulder stiffness is an inflammatory disorder, we thus tried to apply ESWT, an anti-inflammatory modality, in the treatment of rotator cuff lesions with shoulder stiffness. Our study unprecedentedly showed that a single session of high-energy ESWT improves the long-term functional outcome of rotator cuff lesions with shoulder stiffness, suggesting that ESWT is a simple, effective, and noninvasive alternative for the treatment of rotator cuff lesions with shoulder stiffness.

Shock waves are three-dimensional pressure pulses of microsecond duration with the peak pressure of 35–120 million Pa. The focused shock waves are concentrated to a small focal area of 2–8 mm diameter to minimize effects on the surrounding tissues [14]. Different protocols have been proposed for the treatment of shoulder stiffness. Chen et al. applied the shockwave of the energy intensity of 0.6 mJ/mm^2^ to 3 locations (1350 to 1500 shots in each session) at 2-week interval for 3 sessions [32]. We chose a simpler protocol, applying the shockwave of the energy intensity of 0.32 mJ/mm^2^ to subacromial space and rotator interval (3000 shots in each area) for only one session instead and showed comparable results.

The mechanisms of shoulder stiffness included increased expressions of inflammatory cytokines which can induce fibrosis or contracture of subacromial synovium and rotator interval [20, 33, 34]. Lysis of the subacromial adhesions and rotator internal improves the range of motion and functional outcome of the stiff shoulders [5, 12]. We therefore adopted the target areas of subacromial space and rotator interval for the application of ESWT according to the publications mentioned above. In this way, we can avoid the undesired effects of shock wave on the main vasculature to prevent the occurrence of avascular necrosis of the humeral head [35].

Short- to mid-term (3 to 6 months) benefits of ESWT on shoulder disorders have been reported [29, 32, 36]. Our study is the first report to demonstrate the long-term benefits of ESWT in the treatment of rotator cuff lesions with shoulder stiffness.

In our cohort, no significant between-group differences of serum biomarkers were observed before and 1 week and 4 weeks after treatment. The selection of time points is based upon our previous study, showing that the impact of ESWT on systemic biomarkers was most apparent within 4 weeks after intervention [25]. In our previous study, 42 hips with osteonecrosis of femoral head were randomized into three groups. Group A (10 patients, 16 hips) received 2000 impulses of ESWT at 24 kV to the affected hip. Group B (11 patients, 14 hips) and Group C (12 patients, 12 hips) received 4000 and 6000 impulses of ESWT, respectively. The VEGF level in Group C was significantly elevated relative to that of Group A one week after ESWT (*p* = 0.013). Significantly lower IL-6 level in Group C than that in Group A was also noted 1 week after ESWT (*p* = 0.016). Group C showed a significant increase of IGF (*p* = 0.012) relative to Group A 1 month after ESWT [25]. The findings mentioned above were not observed in our study. We hypothesize that fewer impulses (3000 impulses in our study) and different target sites (hip versus shoulder) may account for the discrepancies in the changes of serum biomarkers.

The small sample size was the major limitation of our study. As a result, the separate analysis and comparison between groups based upon the severity of baseline supraspinatus lesion are not allowed. However, the percentage of participants suffering from supraspinatus partial tear, which is more severe than the nontear tendinopathy, was nonsignificantly higher in the ESWT group (42.1%) than in the sham group (22.2%). It is very prudent to suggest that the superior outcome of ESWT is not due to the milder severity of baseline supraspinatus lesion. Our adopted a single session of ESWT with long-term follow-up and good results, suggesting that ESWT is a simple, effective, and noninvasive modality for the treatment of rotator cuff lesions with shoulder stiffness. We believe that these data can be a good reference for further larger scale studies.

## 5. Conclusions

ESWT is a simple, effective, and noninvasive alternative for the treatment of rotator cuff lesions with shoulder stiffness. The benefits of ESWT on the functional outcome can be observed 6 to 12 months after treatment. We hope that these data can become the reference for the therapeutic effects of ESWT on the rotator cuff lesions with shoulder stiffness.

## Figures and Tables

**Figure 1:** The flow chart for the randomizing process.

**Table 1:** Demographic profiles for the two groups.

	ESWT group	Sham group	*p* value
Gender	9 men, 10 women	3 men, 15 women	0.527
Age	52.0 (50.5, 60.5)	51.0 (49.0, 54.0)	0.709
Nontear tendinopathy/partial tear	11/8	14/4	0.197
Subacromial steroid injection^#^	8	7	0.842
Affected shoulder	7 right, 12 left	11 right, 7 left	0.024
Affected shoulder as dominant limb	8 (42.1%)	11 (61.1%)	0.280
BMI	24.5 (21.8, 26.6)	23.1 (22.3, 25.7)	0.688
Medical comorbidities	2 men, 1 woman	0	0.425

BMI: body mass index; ESWT: extracorporeal shockwave therapy. Medical comorbidities included diabetes, coronary artery disease, end-stage renal disease, and liver cirrhosis. ^#^Subacromial steroid injection performed more than 3 weeks before the intervention.

**Table:** (a) Baseline profiles

Outcome	ESWT group	Sham group	*p* value
No. of patients	19	18	
VAS	6.0 (5.0, 7.8)	5.5 (3.3, 7.8)	0.807
Muscle power (lb)	15.0 (14.0, 20.0)	15.0 (13.25, 15.75)	0.089
CMS	44.0 (40.0, 55.0)	44.5 (37.25, 52.25)	0.470

**Table:** (b) One week after intervention

Outcome	ESWT group	Sham group	*p* value
No. of patients	19	18	
VAS	5.0 (4.0, 7.0)	5.5 (3.0, 6.8)	0.640
Muscle power (lb)	16.5 (15.0, 20.75)	15.0 (13.0, 17.0)	0.051
CMS	52.5 (45.5, 60.5)	52.5 (45.0, 58.75)	0.450

**Table:** (c) Four weeks after intervention

Outcome	ESWT group	Sham group	*p* value
No. of patients	19	17	
VAS	5.0 (2.3, 7.0)	3.0 (2.0, 6.0)	0.467
Muscle power (lb)	18.0 (15.0, 20)	16.0 (14.0, 18.0)	0.252
CMS	60.0 (50.5, 71.0)	57.0 (54.0, 67.0)	0.430

**Table:** (d) Three months after intervention

Outcome	ESWT group	Sham group	*p* value
No. of patients	18	15	
VAS	1.0 (0.0, 2.0)	3.0 (1.5, 4.0)	0.089
Muscle power (lb)	18.5 (16.0, 20.0)	16.0 (15.0, 19.0)	0.199
CMS	76.0 (59.0, 82.5)	70.0 (57.5, 72.5)	0.160

**Table:** (e) Six months after intervention

Outcome	ESWT group	Sham group	*p* value
No. of patients	16	15	
VAS	0.0 (0.0, 0.3)	1.0 (0.0, 2.0)	0.012
Muscle power (lb)	20.0 (19.5, 20.0)	18.0 (16.5, 20.0)	0.034
CMS	87.0 (77.5, 91.0)	76.0 (71.3, 78.8)	0.026

**Table:** (f) 12 months after intervention

Outcome	ESWT group	Sham group	*p* value
No. of patients	16	15	
VAS	0.0 (0.0, 0.0)	0.5 (0.0, 2.0)	0.025
Muscle power (lb)	20.0 (20.0, 22.3)	17.5 (16.0, 20.0)	0.002
CMS	91.5 (89.8, 95.0)	85.0 (72.0, 87.0)	0.005

CMS: Constant and Murley score; ESWT: extracorporeal shockwave therapy; VAS: visual analogue scale.

**Table:** (a) Baseline profiles

	ESWT group	Sham group	*p* value
No. of patients	19	18	
Forward flexion (°)	90.0 (85.0, 116.0)	97.5 (90.0, 105.0)	0.940
Abduction (°)	75.0 (67.5, 82.5)	75.0 (70.0, 75.0)	0.196
External rotation (°)	20.0 (15.0, 30.0)	15.0 (15.0, 27.0)	0.787
Internal rotation (°)	15.0 (5.0, 15.0)	15.0 (2.5, 15.0)	0.489
SROM (°)	205.0 (185.0, 247.5)	205.0 (185.0, 227.5)	0.458

**Table:** (b) One week after intervention

	ESWT group	Sham group	*p* value
No. of patients	19	18	
Forward flexion (°)	110.0 (97.5, 120.0)	110.0 (100.0, 120.0)	0.814
Abduction (°)	85.0 (75.0, 100.0)	80.0 (71.25, 90.0)	0.153
External rotation (°)	25.0 (15.0, 30.0)	30.0 (15.0, 43.8)	1.000
Internal rotation (°)	15.0 (3.8, 20.0)	15.0 (10.0, 15.0)	0.703
SROM (°)	240.0 (203.8, 262.5)	235.0 (220.0, 250.0)	0.584

**Table:** (c) Four weeks after intervention

	ESWT group	Sham group	*p* value
No. of patients	19	17	
Forward flexion (°)	120.0 (100.0, 135.0)	120.0 (105.0, 135.0)	0.894
Abduction (°)	100.0 (90.0, 110.0)	90.0 (75.0, 105.0)	0.124
External rotation (°)	30.0 (20.0, 50.0)	40.0 (30.0, 45.0)	0.936
Internal rotation (°)	20.0 (7.5, 30.0)	15.0 (10.0, 30.0)	0.825
SROM (°)	280.0 (232.5, 307.5)	260.0 (240.0, 290.0)	0.483

**Table:** (d) Three months after intervention

	ESWT group	Sham group	*p* value
No. of patients	18	15	
Forward flexion (°)	142.5 (130.0, 157.5)	130.0 (115.0, 140.0)	0.585
Abduction (°)	117.0 (97.5, 127.5)	105.0 (90.0, 110.0)	0.393
External rotation (°)	47.5 (32.5, 68.8)	45.0 (30.0, 55.0)	0.356
Internal rotation (°)	42.5 (22.5, 60.0)	30.0 (17.5, 40.0)	0.039
SROM (°)	347.5 (278.8, 390.0)	305.0 (260.0, 340.0)	0.268

**Table:** (e) Six months after intervention

	ESWT group	Sham group	*p* value
No. of patients	16	15	
Forward flexion (°)	160.0 (145.0, 167.5)	145.0 (135.0, 167.5)	0.397
Abduction (°)	135.0 (120.0, 157.5)	120.0 (110.0, 162.5)	0.486
External rotation (°)	60.0 (60.0, 70.0)	50.0 (40.0, 60.0)	0.012
Internal rotation (°)	60.0 (50.0, 72.5)	45.0 (30.0, 47.5)	<0.001
SROM (°)	430.0 (382.5, 462.5)	365.0 (330.0, 417.5)	0.023

**Table:** (f) 12 months after intervention

	ESWT group	Sham group	*p* value
No. of patients	16	15	
Forward flexion (°)	170.0 (165.0, 175.0)	162.5 (150.0, 175.0)	0.048
Abduction (°)	165.0 (160.0, 170.0)	150.0 (123.8, 170.0)	0.009
External rotation (°)	80.0 (68.8, 81.3)	70.0 (60.0, 75.0)	0.042
Internal rotation (°)	70.0 (60.0, 76.3)	60.0 (51.3, 70.0)	0.031
SROM (°)	485.0 (457.5, 502.5)	445.0 (375.0, 470.0)	0.008

ESWT: extracorporeal shockwave therapy; ROM: range of motion; SROM: sum of range of motion.

**Table:** (a) Baseline profiles

Markers	ESWT group	Sham group	*p* value
IL-6	1.42 (0.97, 2.44)	1.68 (1.24, 2.13)	0.584
TNF-*α*	0.81 (0.71, 1.35)	0.84 (0.53, 1.01)	0.251
IL-1*β*	3.17 (1.96, 5.36)	1.57 (1.00, 3.75)	0.463
TGF-*β*1	26884.6 (21154.3, 29731.4)	24074.3 (20721.7, 28819.6)	0.526
VEFG	168.52 (122.51, 232.54)	163.32 (74.97, 224.38)	0.659
Sub P	176.51 (143.57, 242.21)	167.77 (123.32, 241.10)	0.573
DKK-1	3458.80 (2955.63, 3641.98)	3472.66 (2989.00, 4492.58)	0.322
IGF-1	123.89 (97.99, 157.06)	126.48 (115.47, 149.40)	0.586

**Table:** (b) One week after intervention

Markers	ESWT group	Sham group	*p* value
IL-6	1.32 (1.01, 2.51)	1.58 (1.02, 1.93)	0.690
TNF-*α*	0.84 (0.62, 1.39)	0.75 (0.55, 0.96)	0.131
IL-1*β*	4.61 (1.81, 5.81)	1.05 (0.61, 7.74)	0.525
TGF-*β*1	22324.1 (18882.5, 24578.5)	22404.4 (19687.9, 28536.8)	0.610
VEFG	153.40 (117.70, 209.25)	160.86 (68.38, 195.81)	0.887
Sub P	198.69 (147.02, 240.95)	179.94 (120.48, 318.15)	0.574
DKK-1	3267.62 (2729.97, 3613.64)	3433.46 (2890.84, 4135.69)	0.193
IGF-1	123.72 (99.96, 141.08)	123.46 (106.44, 150.17)	0.518

**Table:** (c) Four weeks after intervention

Markers	ESWT group	Sham group	*p* value
IL-6	1.97 (1.23, 2.73)	1.69 (1.26, 2.11)	0.263
TNF-*α*	0.92 (0.70, 1.41)	0.74 (0.48, 1.18)	0.111
IL-1*β*	3.24 (1.42, 4.79)	1.62 (0.74, 3.39)	0.255
TGF-*β*1	22739.9 (16866.4, 30116.9)	22333.6 (19238.3, 25252.1)	0.568
VEFG	177.68 (107.51, 203.46)	159.75 (72.13, 221.06)	0.947
Sub P	182.28 (160.39, 223.34)	193.86 (130.87, 320.81)	0.681
DKK-1	3449.47 (2915.13, 3825.28)	3281.84 (3008.54, 3939.20)	0.535
IGF-1	132.18 (105.82, 147.21)	138.80 (113.45, 148.44)	0.533

DKK-1: dickkopf-related protein 1; IGF-1: insulin-like growth factor-1; IL-1*β*: interleukin 1-beta; IL-6: interleukin 6; Sub P: substance P; TGF-*β*1: transforming growth factor-beta 1; TNF-*α*: tumor necrosis factor-alpha.

## Data Availability

The data used to support the findings of this study are available from the corresponding author upon request.

## References

[1] Binder A. I., Bulgen D. Y., Hazleman B. L., Roberts S. (1984). Frozen shoulder: a long-term prospective study. *Annals of the Rheumatic Diseases*.

[2] Cofield R. H. (1985). Rotator cuff disease of the shoulder. *The Journal of Bone and Joint Surgery American Volume*.

[3] Ko J. Y., Huang C. C., Chen W. J., Chen C. E., Chen S. H., Wang C. J. (2006). Pathogenesis of partial tear of the rotator cuff: a clinical and pathologic study. *Journal of Shoulder and Elbow Surgery*.

[4] Ozaki J., Fujimoto S., Nakagawa Y., Masuhara K., Tamai S. (1988). Tears of the rotator cuff of the shoulder associated with pathological changes in the acromion. A study in cadavera. *The Journal of Bone & Joint Surgery*.

[5] Ko J. Y., Wang F. S., Huang H. Y., Wang C. J., Tseng S. L., Hsu C. (2008). Increased IL-1beta expression and myofibroblast recruitment in subacromial bursa is associated with rotator cuff lesions with shoulder stiffness. *Journal of Orthopaedic Research*.

[6] Ciampa A. R., de Prati A. C., Amelio E. (2005). Nitric oxide mediates anti-inflammatory action of extracorporeal shock waves. *FEBS Letters*.

[7] Dodenhoff R. M., Levy O., Wilson A., Copeland S. A. (2000). Manipulation under anesthesia for primary frozen shoulder: effect on early recovery and return to activity. *Journal of Shoulder and Elbow Surgery*.

[8] Griesser M. J., Harris J. D., Campbell J. E., Jones G. L. (2011). Adhesive capsulitis of the shoulder: a systematic review of the effectiveness of intra-articular corticosteroid injections. *The Journal of Bone and Joint Surgery American Volume*.

[9] Hsu S. Y., Chan K. M. (1991). Arthroscopic distension in the management of frozen shoulder. *International Orthopaedics*.

[10] Lorbach O., Anagnostakos K., Scherf C., Seil R., Kohn D., Pape D. (2010). Nonoperative management of adhesive capsulitis of the shoulder: oral cortisone application versus intra-articular cortisone injections. *Journal of Shoulder and Elbow Surgery*.

[11] Hsu S. L., Ko J. Y., Chen S. H., Wu R. W., Chou W. Y., Wang C. J. (2007). Surgical results in rotator cuff tears with shoulder stiffness. *Journal of the Formosan Medical Association*.

[12] Ko J. Y., Wang F. S. (2011). Rotator cuff lesions with shoulder stiffness: updated pathomechanisms and management. *Chang Gung Medical Journal*.

[13] Shaffer B., Tibone J. E., Kerlan R. K. (1992). Frozen shoulder. A long-term follow-up. *The Journal of Bone & Joint Surgery*.

[14] Auge B. K., Preminger G. M. (2002). Update on shock wave lithotripsy technology. *Current Opinion in Urology*.

[15] Depalma A. F., Kruper J. S. (1961). Long-term study of shoulder joints afflicted with and treated for calcific tendinitis. *Clinical Orthopaedics*.

[16] Gerdesmeyer L., Wagenpfeil S., Haake M. (2003). Extracorporeal shock wave therapy for the treatment of chronic calcifying tendonitis of the rotator cuff: a randomized controlled trial. *JAMA*.

[17] Ogden J. A., Alvarez R. G., Levitt R., Marlow M. (2001). Shock wave therapy (orthotripsy) in musculoskeletal disorders. *Clinical Orthopaedics and Related Research*.

[18] Speed C. A. (2004). Extracorporeal shock-wave therapy in the management of chronic soft-tissue conditions. *Journal of Bone and Joint Surgery British Volume*.

[19] Wang C. J. (2012). Extracorporeal shockwave therapy in musculoskeletal disorders. *Journal of Orthopaedic Surgery and Research*.

[20] Bunker T. D., Anthony P. P. (1995). The pathology of frozen shoulder. A Dupuytren-like disease. *The Journal of Bone and Joint Surgery British volume*.

[21] Hirschmann M. T., Wind B., Amsler F., Gross T. (2010). Reliability of shoulder abduction strength measure for the Constant-Murley score. *Clinical Orthopaedics and Related Research*.

[22] Gore D. R., Murray M. P., Sepic S. B., Gardner G. M. (1986). Shoulder-muscle strength and range of motion following surgical repair of full-thickness rotator-cuff tears. *The Journal of Bone and Joint Surgery American Volume*.

[23] Constant C. R., Murley A. H. G. (1987). A clinical method of functional assessment of the shoulder. *Clinical Orthopaedics and Related Research*.

[24] Kuo S. J., Wang F. S., Ko J. Y. (2018). Increased expression of type 1 cannabinoid (CB1) receptor among patients with rotator cuff lesions and shoulder stiffness. *Journal of Shoulder and Elbow Surgery*.

[25] Wang C. J., Huang C. C., Yip H. K., Yang Y. J. (2016). Dosage effects of extracorporeal shockwave therapy in early hip necrosis. *International Journal of Surgery*.

[26] Kuo S. J., Hsu H. C., Wang C. J. (2018). Effects of computer-assisted navigation versus conventional total knee arthroplasty on the levels of inflammation markers: a prospective study. *PLoS One*.

[27] Neviaser A. S., Hannafin J. A. (2010). Adhesive capsulitis: a review of current treatment. *The American Journal of Sports Medicine*.

[28] Neviaser A. S., Neviaser R. J. (2011). Adhesive capsulitis of the shoulder. *The Journal of the American Academy of Orthopaedic Surgeons*.

[29] Bannuru R. R., Flavin N. E., Vaysbrot E., Harvey W., McAlindon T. (2014). High-energy extracorporeal shock-wave therapy for treating chronic calcific tendinitis of the shoulder: a systematic review. *Annals of Internal Medicine*.

[30] Frairia R., Berta L. (2011). Biological effects of extracorporeal shock waves on fibroblasts. A review. *Muscles, Ligaments and Tendons Journal*.

[31] Wang C. J., Ko J. Y., Chou W. Y., Cheng J. H., Kuo Y. R. (2018). Extracorporeal shockwave therapy for treatment of keloid scars. *Wound Repair and Regeneration*.

[32] Chen C. Y., Hu C. C., Weng P. W. (2014). Extracorporeal shockwave therapy improves short-term functional outcomes of shoulder adhesive capsulitis. *Journal of Shoulder and Elbow Surgery*.

[33] Bunker T. D., Reilly J., Baird K. S., Hamblen D. L. (2000). Expression of growth factors, cytokines and matrix metalloproteinases in frozen shoulder. *Journal of Bone and Joint Surgery British Volume*.

[34] Rodeo S. A., Hannafin J. A., Tom J., Warren R. F., Wickiewicz T. L. (1997). Immunolocalization of cytokines and their receptors in adhesive capsulitis of the shoulder. *Journal of Orthopaedic Research*.

[35] Liu H. M., Chao C. M., Hsieh J. Y., Jiang C. C. (2006). Humeral head osteonecrosis after extracorporeal shock-wave treatment for rotator cuff Tendinopathy. *The Journal of Bone & Joint Surgery*.

[36] Galasso O., Amelio E., Riccelli D. A., Gasparini G. (2012). Short-term outcomes of extracorporeal shock wave therapy for the treatment of chronic non-calcific tendinopathy of the supraspinatus: a double-blind, randomized, placebo-controlled trial. *BMC Musculoskeletal Disorders*.

